The article "Evaluation of Pakistani wheat germplasm for leaf rust resistance at various locations" was retracted in 2022. Reasons: compromised peer review; a conflict of interest; concerns about the authorship.

# Evaluation of Pakistani wheat germplasm for leaf rust resistance at various locations

**DOI:** 10.1371/journal.pone.0266695

**Published:** 2022-05-04

**Authors:** Sabina Asghar, Aziz Ur Rehman, Nadeem Ahmad, Sadia Ajmal, Aneela Ahsan, Saima Gulnaz, Makky Javed, Javed Ahmad, Javed Iqbal, Sumera Bibi, Sajid Fiaz, Basem H. Elesawy, Ahmad El Askary, Khadiga Ahmed Ismail, Amal F. Gharib, Ahsan Mohyo-ud-Din, Muhammad Ijaz Tabassum, Abdul Qayyum

**Affiliations:** 1 Wheat Research Institute, Ayub Agriculture Research Institute, Faisalabad, Pakistan; 2 Wheat Breeding Section, Barani Agricultural Research Institute, Chakwal, Pakistan; 3 Department of Environmental Sciences, COMSATS University Islamabad, Abbottabad Campus, Abbottabad, Pakistan; 4 Department of Plant Breeding & Genetics, The University of Haripur, Haripur, Pakistan; 5 Department of Pathology, College of Medicine, Taif University, Taif, Saudi Arabia; 6 Department of Clinical Laboratory Sciences, College of Applied Medical Sciences, Taif University, Taif, Saudi Arabia; 7 Oilseed Research Institute, Ayub Agriculture Research Institute, Faisalabad, Pakistan; 8 Department of Agronomy, The University of Haripur, Haripur, Pakistan; Anhui Agricultural University, CHINA

## Abstract

341 entries comprising of 250 genotypes/lines and 91 gene differentials were tested for leaf rust (*Puccinia triticina* Erik) in different ecological zones of Punjab during 2016–17 and 2017–18. Each entry was planted in a single 1 m long row and Morocco was used as a spreader. Data on leaf rust severity was recorded once in 3^rd^ week of March during both study years at all locations by following Modified Cobb Scale while the data was recorded three times on 2^nd^, 22^nd^ and 29^th^ March during 2018 at Faisalabad location to study rust development pattern. The disease severity ranged from 0-100S during 2016–17 and from 0-80S during 2017–18. The genotype HYT 60–5 and the genes *Lr*-19, *Lr*-26 and *Lr* 27+31 showed no disease symptoms at any location during both the study years. These genes can be used for future breeding material development. Area under disease progressive curve (AUDPC), calculated on the basis of periodical readings from Faisalabad, ranged from 0–550 and the susceptible check Morocco has AUDPC value of 600. 120 entries including HYT 60–5 have disease progression 0, which showed that there may be a major gene based resistance in these entries. Area under disease progressive curve/Day (AUDPC/DAY) was calculated for the rest of 130 genotypes to have an understanding of the disease progression pattern and out of which 43 entries have AUDPC/Day value ranging from 1–2 and 28 entries have AUDPC/Day value ranging from 2–3 which revealed that these entries are very useful for use in breeding for durable rust resistance and can be utilized as a parent in back cross and top cross breeding schemes. Material with AUDPC value less than 10 is the best source of resistance against the leaf rust. Varieties/advanced lines, Ujala-16, V-14154, and V-14124 have shown slow rust development and are very good sources of resistance. Similarly, HYT 60–5 has proven an excellent source of resistance. The advance line V-14154 has been approved as a commercial cultivar by the name “Akbar-19”.

## Introduction

Wheat is one of the most important cereals in the world. Since green revolution, there is many fold increase in wheat production especially in the developing world [1]. Many factors are responsible for limiting wheat production like heat stress, drought stress, diseases and insect pests etc. Among different diseases like bunts, rusts and other foliar diseases rusts have induced serious yield losses [2].

Chemical control of the rust is being practiced in developed countries whereas in the developing world, it is not affordable for the farmers. Hence, they depend upon genetic resistance [3, 4] and development of resistant cultivars is considered the most effective way to manage the disease [5, 6]. Identification of genetic variability for rust resistance and its use to develop resistant cultivars through schematic breeding is pre-requisite to develop rust resistant cultivars. During the post green revolution period, cultivars with different genes (*Lr10*, *Lr13*, *Lr26* etc) have continuously been released across the world and eliminated with the passage of time [4, 7, 8].

Leaf rust caused by *Puccina triticina* is a serious threat and results in major yield losses to wheat production in temperate zone areas like Pakistan where climate is generally arid, characterized by hot summers and cool or cold winters and wide variations between extremes of temperature at given locations [9]. Wheat breeders mostly introduced wheat breeding material mostly depending upon varieties containing genes *Lr 1*, *Lr 13 and Lr 26* in combination with the minor genes [4]. These varieties help to boost up wheat production due to higher yield potential and adaptability to rusts especially for leaf rust resistance. However due to emergence of new leaf rust races in a short time period, the breeders periodically deployed new rust resistance genes all over the world [10]. The resistance of cultivars developed with monogenic or vertical résistance is not durable, therefore now, the breeders are mainly depending on new sources of resistance to leaf rust based on minor genes which slows down the rust development and significantly reduce the losses due to rusts [11]. Breeders are looking for the genotypes with slow rusting mechanism for use in the breeding program. In previous years, many accessions with this type of resistance have been selected [12–14] and were used for developing back crosses, top crosses for pyramiding minor genes present in wheat germplasm [15] and many wheat varieties like Seher-06, Shafaq-06, Lasani-08, Faisalabad-08, AARI-11, Pb-11, Galaxy-13 etc have been released which contributed significantly in enhancing wheat production in the Punjab province and were cultivated in other provinces of Pakistan [4, 16, 17]. Breeders are now preferring genotypes with slow rusting or horizontal resistance based on minor genes or combination of minor and major genes [8, 18]. Area Under Disease Progressive Curve (AUDPC) has been used by many scientists to understand disease development pattern and they preferred the genotypes having slow rusting pattern with lower AUDPC values for disease [19]. The current studies were designed to evaluate wheat germplasm for identification of sources of leaf rust resistance, to identify the resistance mechanism and pattern of rust development.in different ecological zones of Punjab- Pakistan.

## Materials and methods

### i-Experimental material & locations

A set of germplasm comprising of 341 entries (250 varieties/advanced lines of local origin and 91 genes differential received from CIMMYT, Mexico) were sown in the 3^rd^ week of November during the years 2016–17 and 2017–18 at four different locations of Punjab viz. Wheat Research Institute, Faisalabad (31.4504° N and 73.1350° E, Punjab Seed Corporation, Khanewal (30.2864° N and 71.9320° E), Regional Agriculture Research Institute, Bahawalpur (29.3544° N and 71.6911° E) and Agriculture Adaptive Research Farm, Kot Naina district Narowal (32.1836° N and 75.2523° E) which were located in different agro-ecological zones of the Punjab having difference in temperature and rainfall pattern (Table 1).

**Table 1:** Historical (2010–2020) average maximum temperature, average minimum temp and average rainfall of experimental sites during wheat growing season (worldweatheronline.com).

Months	Kot Naina			Faisalabad			Khanewal			Bahawalpur		
	Max °C	Min °C	Rainfall (mm)	Max °C	Min °C	Rainfall (mm)	Max °C	Min °C	Rainfall (mm)	Max °C	Min °C	Rainfall (mm)
November	28	16	20.7	30	18	3.3	31	18	1.4	31	19	1.5
December	23	11	36.4	25	15	3.4	25	13	3.4	26	15	3.5
January	20	9	54.4	27	10	17.2	23	11	8.6	23	13	3.4
February	23	11	93.0	25	12	28.0	26	13	12.5	27	15	6.9
March	29	15	88.8	31	16	34.6	32	17	17.0	33	20	13.3

### ii-Experiment management

Each entry was sown in a 2 m long single row by maintaining 30 cm row to row distance. A single line of susceptible cultivar, Morocco was repeatedly sown after every 10lines of experimental material. Two rows of spreader “Morocco” were sown on each side of the experimental material to capture pathotype inoculum. The fertilizer NPK was applied as a basil dose at the rate of 120, 75 and 60 kg ha^-1^. Three irrigations were applied at different growth stages i.e. first at tillering stage, second at booting stage and third at grain formation stage. Weeds were controlled by manual hoeing at all four locations.

### iii-Inoculation of experimental material

The inoculation of material was done three times during first fortnight of February at an interval of five days at all locations. The previous years collected inoculums mixture (mixture of pathotypes found from all over Punjab) stored at -80°C was used after proper heat shock and re-hydration process. 1 g of inoculum was mixed in 250 g of talcum powder and was dusted on experimental material.

### iv-Data recording and analysis

At Faisalabad during the year 2017–2018, the leaf rust data was recorded three times at two-week interval starting from 01-03-2018 to 29-03-2018. The data was used to calculate Area Under Disease Progressive Curve (AUDPC) [20–22]. The AUDPC was calculated by using Excel based software developed by CIMMYT [20].

$$\text{AUDPC}=\overset{\text{n}}{\underset{i=1}{\sum }}[\left\{(Y_{i}+Y_{\left(i+1\right)})/2\}\;\text{x}\;(t_{\left(i+1\right)}-t_{i}\right)]$$

Where Y_i_ is disease severity at t_i_ time, *t*_(*i*+1)_ − *t*_*i*_ is time interval between two consecutive data recording events, n is no. of data recordings.

AUDPC/Day was calculated by dividing AUDPC with the number of days counted from the first to the last data recording date. At all other three locations except, disease appearance was based on natural inoculation. The data was recorded once during 4^th^ week of March. The data was recorded following Modified Cobb’s Scale and the entries were classified as resistant, moderately resistant, moderately susceptible, moderately resistant to moderately susceptible and susceptible [23].

## Results

Screening of wheat germplasm for leaf rust resistance is a constant feature of our research program. In the current study, a set of 341 genotypes comprising of 250 varieties/advanced lines and 91 gene differentials were evaluated against leaf rust in field conditions. Tables 2–6 shows reaction of this set of genotypes to leaf rust at four locations viz. Faisalabad, Bahawalpur, Khanewal and Kot Naina during the study years.

**Table 2:** Leaf rust reactions, symbol, field response and value of response.

Reaction	Symbol	Field Response
No disease	0	No visible infection
Resistant	R	Necrotic area with or without minute uredia
Moderately resistant	MR	Small uredia present surrounded by necrotic area
Moderately susceptible	MS	Medium uredia with no necrosis but some distinct chlorosis.
Moderately resistant moderately susceptible	MRMS	Small uredia present surrounded by necrotic areas as well as medium uredia with no necrosis but some distinct chlorosis.
Susceptible	S	Large uredia and little or no chlorosis present.

**Table 3:** Leaf rust resistant genotypes during 2016–17 at different locations.

Reaction	Faisalabad			Bahawalpur			Khanewal			KotNaina		
	No of genotypes	lines/ varieties	Gene differentials	No of genotypes	lines/ varieties	Gene differentials	No of genotypes	lines/ varieties	Gene differentials	No of genotypes	lines/ varieties	Gene differentials
No disease	17	15235, 60–5	Lr-19, Lr -26, Lr-27+31, Yr-1, Yr-9, Yr-10, Yr-15, Yr-24, Sr-5, Sr-6, Sr-7A, AOC-YRA, AOC+YRA, SRGP, SRAC-1	30	15235, 60–5, TATARA, Ujalla-16	Lr -9, Lr -18, Lr-19, Lr-22A, Lr-26, Lr-27+31, Lr-36, Yr-1, Yr-2, Yr-5, Yr-6, Yr-7, Yr-9, Yr-10, Yr-15, Yr-17, Yr-18, Yr-24, Yr-CV, Sr-5, Sr-6, Sr-7A, AOC-YRA, AOC+YRA, SRGP, SRAC-1	32	15235, 60–5, TATARA, Ujalla-16	Lr-9, Lr -18, Lr-19, Lr-22A, Lr-26, Lr-27+31, Lr-28, Lr- 36, Yr-1, Yr-2, Yr-5, Yr-6, Yr-7, Yr-9, Yr-10, Yr-15, Yr-17, Yr-18, Yr-24, Yr-26, Yr-CV, Sr-5, Sr-6, Sr-7A, AOC-YRA, AOC+YRA, SRGP, SRAC-1	58	14124, 14154, 15235, 60–5, 60–57, WL-711, TATARA, PBW-343, SERI, SUPER KAUZ, Ujalla-16, Galaxy-13, Pb-11, AARI-11, Millat-11, Fsd-08, Lasani-08, Seher-06, Inq-91	Lr-9, Lr-12, Lr-13, Lr-15, Lr-16, Lr-17, Lr-18, Lr-19, Lr-21, Lr-22A, Lr-25, Lr-26, Lr- 27+31, Lr-36, Lr-23+GAZA, Yr-1, Yr-2, Yr-5, Yr-6, Yr-7, Yr-9, Yr-10, Yr-15, Yr-17, Yr-18, Yr-24, Yr-26, Lr-27, Lr-28, Yr-29, Yr-31, Yr-CV, Sr-5, Sr-6, Sr-7A, AOC-YRA, SRGP, SRAC-1, AOC+YRA
Resistant	6	-	Lr-18, Lr-22A, Lr-36, Yr-CV, Yr-7, Yr-26	-	-	-	-	-	-	2	-	Lr-22B, Lr-B
Moderately resistant	1	-	Lr-23+GAZA	3	-	Lr-23+GAZA, Yr-26, YR-28	1	-	Lr-23+GAZA	-	-	-
Moderately resistant-moderately susceptible	15	14124, 14154, PBW-343, Ujalla-16, Pb-11, Millat-11, Fsd-08	Lr-16, Lr-22B, Lr-23, Lr-25, Lr-28, Yr-5, YR-18, Yr-28	10	14124, 14154, PBW-343, Pb-11, Millat-11, Fsd-08	Lr-16, Lr-22B, Lr-23, Lr-28	9	14154, PBW-343, Pb-11, Millat-11, Fsd-08	Lr-16, Lr-22B, Lr-23, Yr-28	1	-	Lr-35
Moderately susceptible	4	60–57, Inq-91	Lr-29, Lr-33	3	60–57	Lr-29, Lr-33	3	14124	Lr-29, Lr-33	1	-	Lr-29
Susceptible	32	WL-711, TATARA, SERI, SUPER KAUZ, Galaxy-13, AARI-11, Lasani-08, Seher-06	Lr-9, Lr-10, Lr-11, Lr-12, Lr-13, Lr-14A, Lr-14B, Lr-15, Lr-17, Lr-20, Lr-21, Lr-24, Lr-30, Lr-32, Lr-34, Lr-35, Lr-37, Lr-B, Yr-2, Yr-6, Yr-17, Yr-27, Yr-29, Yr-31	29	WL-711, SERI, SUPER KAUZ, Galaxy-13, AARI-11, Lasani-08, Seher-06, Inq-91	Lr-10, Lr-11, Lr-12, Lr-13, Lr-14A, Lr-14B, Lr-15, Lr-17, Lr-20, Lr-21, Lr-24, Lr-25, Lr-30, Lr-32, Lr-34, Lr-35, Lr-37, Lr-B, Yr-27, Yr-29, Yr-31	29	WL-711, SERI, SUPER KAUZ, Galaxy-13, AARI-11, Lasani-08, Seher-06, Inq-91	Lr-10, Lr-11, Lr-12, Lr-13, Lr-14A, Lr-14B, Lr-15, Lr-17, Lr-20, Lr-21, Lr-24, Lr-25, Lr-30, Lr-32, Lr-34, Lr-35, Lr-37, Lr-B, Yr-27, Yr-29, Yr-31	7	-	Lr-10, Lr-11, Lr-14B, Lr-24, Lr-30, Lr-34, Yr-6

**Table 4:** Genotypes resistant to leaf rust at all locations during 2016–17.

Reaction	Faisalabad			Bahawalpur			Khanewal			KotNaina		
	No of genotypes	lines/ varieties	Gene differentials	No of genotypes	lines/ varieties	Gene differentials	No of genotypes	lines/ varieties	Gene differential	No of genotypes	lines/ varieties	Gene differentials
No disease	17	15235, 60–5	Lr-19, Lr-26, Lr-27+31, Yr-1, Yr-9, Yr-10, Yr-15, Yr-24, Sr-5, Sr-6, Sr-7A, AOC-YRA, AOC+YRA, SRGP, SRAC-1	17	15235, 60–5	Lr-19, Lr-26, Lr-27+31, Yr-1, Yr-9, Yr-10, Yr-15, Yr-24, Sr-5, Sr-6, Sr-7A, AOC-YRA, AOC+YRA, SRGP, SRAC-1	17	15235, 60–5	Lr-19, Lr-26, Lr-27+31, Yr-1, Yr-9, Yr-10, Yr-15, Yr-24, Sr-5, Sr-6, Sr-7A, AOC-YRA, AOC+YRA, SRGP, SRAC-1	17	15235, 60–5	Lr-19, Lr-26, Lr-27+31, Yr-1, Yr-9, Yr-10, Yr-15, Yr-24, Sr-5, Sr-6, Sr-7A, AOC-YRA, AOC+YRA, SRGP, SRAC-1
Resistant	-	-	-	-	-	-	-	-	-	-	-	-
Moderately resistant	-	-	-	-	-	-	-	-	-	-	-	-
Moderately resistant-moderately susceptible	-	-	-	-	-	-	-	-	-	-	-	-
Moderately susceptible	1	-	Lr-29	1	-	Lr-29	1	-	Lr-29	1	-	Lr-29
Susceptible	6	-	Lr-10, Lr-11, Lr-14B, Lr-24, Lr-30, Lr-34	6	-	Lr-10, Lr-11, Lr-14B, Lr-24, Lr-30, Lr-34	6	-	Lr-10, Lr-11, Lr-14B, Lr-24, Lr-30, Lr-34	6	-	Lr-10, Lr-11, Lr-14B, Lr-24, Lr-30, Lr-34

**Table 5:** Leaf rust resistant genotypes during 2017–18 at different locations.

Reaction	Faisalabad			Bahawalpur			Khanewal			KotNaina		
	No of genotypes	lines/ varieties	Gene differentials	No of genotypes	lines/ varieties	Gene differentials	No of genotypes	lines/ varieties	Gene differentials	No of genotypes	lines/ varieties	Gene differentials
No disease	22	60–5, Ujalla-16	Lr-19, Lr-26, Lr-27+31, Lr- 36, Lr-23+GAZA, Yr-1, Yr-5, Yr-7, Yr-10, Yr-24, Yr-26, Yr-29, Yr-31, Yr-CV, Sr-5, Sr-6, AOC-YRA, AOC+YRA, SRGP, SRAC-1,	58	14124, 14154, 15235, 60–5, 60–57, TATARA, PBW-343, SERI, SUPER KAUZ, Ujalla-16, Pb-11, Millat-11	Lr-9, Lr-10, Lr-11, Lr-12, Lr-13, Lr-14A, Lr-14B, Lr-15, Lr-16, Lr-17, Lr-18, Lr-19, Lr-21, Lr-22B, Lr-23, Lr-24, Lr-26, Lr- 27+31, Lr-28, Lr-29, Lr-36, Lr-23+GAZA, Yr-1, Yr-2, Yr-5, Yr-6, Yr-7, Yr-9, Yr-10, Yr-15, Yr-17, Yr-18, Yr-24, Yr-26, Lr-27, Lr-28, Yr-29, Yr-31, Yr-CV, Sr-5, Sr-6, Sr-7A, AOC-YRA, AOC+YRA, SRGP, SRAC-1	69	14124, 14154, 15235, 60–5, 60–57, WL-711, TATARA, PBW-343, SERI, SUPER KAUZ, Ujalla-16, Galaxy-13, Pb-11, AARI-11, Millat-11, Lasani-08, Inq-91	Lr-9, Lr-10, Lr-11, Lr-12, Lr-14A, Lr-14B, Lr-15, Lr-16, Lr-17, Lr-18, Lr-19, Lr-21, Lr-22A, Lr-22B, Lr-23, Lr-24, Lr-26, Lr-27+31, Lr-28, Lr-29, Lr-30, Lr-33, Lr-34, Lr-35, Lr-36, Lr-37, Lr-B, Lr-23+GAZA, Yr-1, Yr-2, Yr-5, Yr-6, Yr-7, Yr-9, Yr-10, Yr-15, Yr-17, Yr-18, Yr-24, Yr-26, Lr-27, Lr-28, Yr-29, Yr-31, Yr CV, Sr-5, Sr-6, Sr-7A, AOC-YRA, AOC+YRA, SRGP, SRAC-1	75	14124, 14154, 15235, 60–5, 60–57, WL-711, TATARA, PBW-343, SERI, SUPER KAUZ, Ujalla-16, Galaxy-13, Pb-11, AARI-11, Millat-11, Fsd-08, Lasani-08, Seher-06, Inq-91	Lr-9, Lr-10, Lr-11, Lr-12, Lr-13, Lr-14A, Lr-14B, Lr-15, Lr-16, Lr-17, Lr-18, Lr-19, Lr-20, Lr-21, Lr-22A, Lr-22B, Lr-23, Lr-24, Lr-25, Lr-26, Lr-27+31, Lr-28, Lr-29, Lr-30, Lr-32, Lr-33, Lr-34, Lr-35, Lr-36, Lr-37, Lr- B, Lr-23+GAZA, Yr-1, Yr-2, Yr-5, Yr-6, Yr-7, Yr-9, Yr-10, Yr-15, Yr-17, Yr-18, Yr-24, Yr-26, Lr-27, Lr-28, Yr-29, Yr-31, Yr CV, Sr-5, Sr-6, Sr-7A, AOC-YRA, AOC+YRA, SRGP, SRAC-1,
Resistant	-	-	-	-	-	-	-	-	-	-	-	-
Moderately resistant	1	Pb-11	-	1	-	Lr-20	-	-	-	-	-	-
Moderately resistant-moderately susceptibl	5	14124, 14154, 60–57, PBW-343, SUPER KAUZ	-	-	-	-	-	-	-	-	-	-
Moderately susceptible	19	15235, SERI, AARI-11, MILLAT-11, FSD-08, LASANI-08	Lr-10, Lr-11, Yr-18, Yr-27, Yr-28, SR-7A, Lr-24, Lr-29, Lr-30, Yr-18, Yr-27, Yr-28, SR-7A	10	AARI-11, FSD-08, LASANI-08	Lr-25, Lr-30, Lr-33, Lr-34, Lr-35, Lr-37, Lr-B	6	FSD-08, SEHER-06	Lr-13, Lr-22A, Lr-25, Lr-32	-	-	-
Susceptible	31	TATARA, Galaxy-13, Seher-06, Inq-91	Lr-9, Lr-12, Lr-13, Lr-14A, Lr-14B, Lr-15, Lr-16, Lr-17, Lr-18, Lr-20, Lr-21, Lr-22A, Lr-22B, Lr-23, Lr-25, Lr-28, Lr-32, Lr-33, Lr-34, Lr-35, Lr-37, Lr-B, Yr-2, Yr-6, Yr-9, Yr-15, Yr-17	5	WL-711, Galaxy-13, Seher-06, Inq-91	Lr-32	1	-	Lr-20	-	-	-

**Table 6:** Genotypes resistant to leaf rust at all locations during 2017–18.

Reaction	Faisalabad			Bahawalpur			Khanewal			KotNaina		
	No of genotypes	lines/ varieties	Gene differentials	No of genotypes	lines/ varieties	Gene differentials	No of genotypes	lines/ varieties	Gene differentials	No of genotypes	lines/ varieties	Gene differentials
No disease	22	60–5, Ujalla-16	Lr-19, Lr-26, Lr-27+31, Lr- 36, Lr-23+GAZA, Yr-1, Yr-5, Yr-7, Yr-10, Yr-24, Yr-26, Yr-29, Yr-31, Yr-CV, Sr-5, Sr-6, AOC-YRA, AOC+YRA, SRGP, SRAC-1,	22	60–5, Ujalla-16	Lr-19, Lr-26, Lr-27+31, Lr- 36, Lr-23+GAZA, Yr-1, Yr-5, Yr-7, Yr-10, Yr-24, Yr-26, Yr-29, Yr-31, Yr- CV, Sr-5, Sr-6, AOC-YRA, AOC+YRA, SRGP, SRAC-1	22	60–5, Ujalla-16	Lr-19, Lr-26, Lr-27+31, Lr- 36, Lr-23+GAZA, Yr-1, Yr-5, Yr-7, Yr-10, Yr-24, Yr-26, Yr-29, Yr-31, Yr- CV, Sr-5, Sr-6, AOC-YRA, AOC+YRA, SRGP, SRAC-1	22	60–5, Ujalla-16	Lr-19, Lr-26, Lr- 27+31, Lr-36, Lr-23+GAZA, Yr-1, Yr-5, Yr-7, Yr-10, Yr-24, Yr-26, Yr-29, Yr-31, Yr-CV, Sr-5, Sr-6, AOC-YRA, AOC+YRA, SRGP, SRAC-1
Resistant	-	-	-	-	-	-	-	-	-	-	-	-
Moderately resistant	-	-	-	-	-	-	-	-	-	-	-	-
Moderately resistant-moderately susceptible	-	-	-	-	-	-	-	-	-	-	-	-
Moderately susceptible	-	-	-	-	-	-	-	-	-	-	-	-
Susceptible	-	-	-	-	-	-	-	-	-	-	-	-

### i-1^st^ year results

During the year 2016–2017, there was no disease reaction on 17 entries (Table 3) at Faisalabad. Out of these, 2 were the advanced lines and remaining 15 were gene differentials. Similarly, there was no disease on 30 entries containing 2 advanced lines and 2 approved varieties. At Khanewal, there was no disease on 4 advanced lines, approved varieties and 28 gene differentials. At Kot Naina, disease did not appear on 58 entries and out of these, 19 were advanced lines/varieties and 39 were gene differentials. The differences in the response of different genotypes at different locations might be due to variation in environmental conditions as shown in Table 1 and variation in the natural inoculum prevailing at these locations. Two advanced lines V-15235 and HYT 60–5 and fifteen gene differentials did not show any disease symptoms whereas one gene differential *Lr-29* was moderately susceptible on all four locations of Punjab, Pakistan during the year 2016–17 (Table 4). 6 gene differentials (*Lr-10*, *Lr-11*, *Lr-14B*, *Lr-24*, *Lr-30 and Lr-34*) showed susceptibility.

### ii-2^nd^ year results

During the year 2017–2018, there was no disease appeared on 2 genotypes HYT 60–5 and Ujala-16 whereas 28 differentials were free from leaf rust at Faisalabad (Table 5). At Bahawalpur, 58 entries did not show any disease reaction and out of these 12 were advanced lines/varieties and rests were the gene differentials. At Khanewal, 69 entries were disease free. Among these 69, 17 were advanced lines/varieties and 52 were gene differentials. At Kot Naina, 75 entries were completely free from leaf rust disease. Out of these, 18 were advanced lines/varieties and remaining were gene differentials. A variety Punjab-11 at Faisalabad and gene *Lr*-20 at Bahawalpur showed moderately resistant behavior. The advanced lines/varieties V-14124, V-14154, V-HYT 60–57, PBW-343 and SUPER KAUZ showed moderately resistant to moderately susceptible reaction at Faisalabad.

During the year 2017–2018, 22 entries were common in the entries containing 1 advanced line V-HYT 60–5 and 1 variety Ujala-16 and gene differentials (Table 6). 1 advanced line V-HYT 60–5 and 1 variety Ujala-16 and the gene differentials i.e. *Lr 19*, *Lr 26*, *Lr 27+31*, *Lr 36*, *Lr 23+GAZA*, *Yr-1*, *Yr-5*, *Yr-7*, *Yr-10*, *Yr-24*, *Yr-26*, *Yr-29*, *Yr-31*, *Yr CV*, *Sr-5*, *Sr-6*, AOC-YRA, AOC+YRA, SRGP, SRAC-1 did not show any disease reaction at all four locations of Punjab, Pakistan.

### iii-Future sources of resistance

The advance line HYT 60–5 had not shown disease symptom at any experimental location during both the study years (Table 7) in Punjab, Pakistan. Therefore, this can be treated as the most promising leaf rust resistant genotype for use in the breeding program. Similarly, the leaf rust gene differentials containing *Lr-19*, *Lr-26 and Lr-27+31* genes did not show any susceptibility at any target location during both study years. Therefore, the material containing these 3 genes may be targeted for improving leaf rust resistance in bread wheat breeding material.

**Table 7:** Common leaf rust resistant genotypes at all locations during both years 2016–17 and 2017–18.

Reaction	Faisalabad			Bahawalpur			Khanewal			KotNaina		
	No of genotypes	lines/ varieties	Gene differentials	No of genotypes	lines/ varieties	Gene differentials	No of genotypes	lines/ varieties	Gene differentials	No of genotypes	lines/ varieties	Gene differentials
No disease	13	60–5	Lr--19, Lr-26, Lr-27+31, Yr-1, Yr-10, Yr-24, Sr-5, Sr-6, AOC-YRA, AOC+YRA, SRGP, SRAC-1	13	60–5	Lr--19, Lr-26, Lr-27+31, Yr-1, Yr-10, Yr-24, Sr-5, Sr-6, AOC-YRA, AOC+YRA, SRGP, SRAC-1	17	60–5	Lr-19, Lr-26, Lr-27+31, Yr-1, Yr-10, Yr-24, Sr-5, Sr-6, AOC-YRA, AOC+YRA, SRGP, SRAC-1	17	60–5	Lr-19, Lr-26, Lr-27+31, Yr-1, Yr-10, Yr-24, Sr-5, Sr-6, AOC-YRA, AOC+YRA, SRGP, SRAC-1
Resistant	-	-	-	-	-	-	-	-	-	-	-	-
Moderately resistant	-	-	-	-	-	-	-	-	-	-	-	-
Moderately resistant-moderately susceptible	-	-	-	-	-	-	-	-	-	-	-	-
Moderately susceptible	-	-	-	-	-	-	-	-	-	-	-	-
Susceptible	-	-	-	-	-	-	-	-	-	-	-	-

### iv-Disease progression

Area under disease progression curve (AUDPC) show disease development in relation to time period and AUDPC/Day gives its clear picture. In the present study during the year 2017–18, AUDPC was calculated to find out disease progression pattern. AUDPC ranged from 0–550 while that of Morocco which is a susceptible check has AUDPC value of 600. 120 entries have disease progression 0 which shows there may be a major gene-based resistance in these entries. AUDPC/Day was calculated for the rest of 130 entries to have a deep understanding of the disease progression and out of which 43 entries have AUDPC/Day value ranging from 1–2 and 28 entries have AUDPC/Day value ranging from 2–3. These entries have slow rust development pattern than average which shows that these entries are extremely useful for use in breeding for durable rust resistance and can be utilized as a parent in back cross and top cross in breeding scheme.

## Discussion

In Past, wheat varieties with different types of rust resistance mechanism have been released all over the world including Pakistan [24, 25]. The varieties having monogenic and varietal resistance generally have short life whereas the varieties with multiple gene resistance and horizontal resistance have long life [1, 11, 14, 15]. Furthermore, use of monogenic resistance also sometimes create monocentric situation. Material possessing 1B-1R translocation was used all over the world and results in the evolution of new devastating genes like *Yr 9*, *Yr 27* and Ug99 [4, 6, 9]. Current studies revealed that most of the gene differentials studied showed virulence however virulence for *Lr 19*, *Lr 26 and Lr 27+31* was not present in the Punjab, Pakistan. Therefore, the varieties having adult plant resistance based on minor genes were preferred by wheat breeders [4, 12]. Among the advanced lines/varieties tested, only one entry HYT 60–5 has not shown any disease symptoms which might be due to the presence of major gene and combination of major/minor gene. Advanced lines V-14124, V-14154, V-15235 and HYT 60–57 have shown no disease development at Bahawalpur, Khanewal and Kot Naina where disease inoculation was not applied. However, V-14124, V-14154 and HYT 60–57 showed moderately resistant reaction whereas V-15235 showed moderately susceptible reaction during 2017–18. In 2016–17, the line V-15235 has not shown any disease symptoms at Faisalabad, Bahawalpur, Kala Shah Kaku and Kot Naina whereas the lines V-14124 and V-14154 showed moderately resistant reaction which shows that these lines have horizontal resistance based on minor genes. V-14154 has been approved as Akbar-19 due to its better performance in yield trials and disease screening nurseries at national level [25]. Presence of minor genes-based resistance has been reported in international and Pakistani germplasm by [15, 26]. During 2017–18, there was no disease on HYT 60–5. Among approved wheat varieties, Ujala-16 has not shown any disease during 2017–18 whereas at Bahawalpur, Khanewal and Kot Naina, it showed moderately resistant moderately susceptible (MRMS) reaction. Variable disease reactions of different wheat genotypes have already been reported in literature due to different genetic background of breeding material and variation in environmental conditions [8, 16].

As far as reaction of gene differentials is concerned, leaf rust resistant genes *Lr19*, *Lr26*, *Lr 27+31* have not shown any virulence. Therefore, these genes can be used as a source of leaf rust resistance in wheat breeding program preferably in combination with other major and minor genes because it has been revealed that the cultivars having major and minor gene combinations have high and sustainable level of resistance which showed that variation in the disease progression level is due to the difference in host pathogen interaction [18].

Area under disease progressive curve (AUDPC) values ranged from 0 to 690. Maximum AUDPC was recorded in case of susceptible universal check, Morocco. AUDPC/Day was calculated by dividing AUDPC with the number of days. The range for AUDPC/Day ranged from 0–25 with the average value of 4.72. There are 122 genotypes which have shown AUDPC/Day value of 0 and 92 genotypes fall in the AUDPC/Day values range from 1–5. 14 genotypes have shown AUDPC/Day value ranging from 6–10. 7 genotypes have AUDPC/Day value in the range of 11–15. There are 6 genotypes showing AUDPC/Day value ranging from 16–20 and 36 genotypes having AUDPC/Day value above 20 (Table 8). AUDPC/Day value is the indicator of progression rate. The genotypes with lower AUDPC value have lesser disease development rate as compared to the genotypes with higher AUDPC/Day value. It was concluded that the genotypes having AUDPC/Day value less than 10 can be utilized as valuable source in the breeding program and such material with lower AUPDC values can be released for commercial cultivation as use of such material is environment friendly, enhances farmers profitability.

**Table 8:** Classification of advanced lines on the basis of area under disease progressive curve.

AUDPC/Day Value	No. of genotypes	Genotypes
0	120	60–5, 15082, 15099, 16005, 15113, 15291, 15166, 15216, 1038, 14058, 14061, 20–6, 20–19, 55–33, NS-76, 15–29, 1432, 1578, 1579, 1581, 15–1711, 15–1713, 15–1725, 15–1755, 16-CO38, 16-CO39, NR-521, NR-523, NR-525, 15 BT 001, NW-2-17, Morocco, Ujala-16, Chak-50, Pb-76, Pavon-76, 16222, 16227, 16233, 16259, 16261, 16266, 16274, 16275, 16276, 16277, 16287, 16289, 16282, 16280, 16265, 16290, 16291, 16293, 16294, 16295, 16221, 16260, 16003, 16004, 16005, 16006, 16018, 16023, 16024, 16025, 16036, 16049, 16051, 16077, 16079, 16087, 16090, 16124, 16125, 16128, 16129, 16131, 16132, 16134, 16144, 16145, 16146, 16147, 16152, 16153, 16157, 16150, 16160, 17153, 17154, 17155, 17157, 17158, 17159, 17161, 17162, 17163, 17165, 17169, 17170, 17171, 17175, 17176, 17177, 17180, 17182, 17183, 16106, 16108, 16111, 15012, 15009, 5011, 15018, 15035, 15006, 14003, 14011, 14035.
1–2	43	14124, 14154, 15070, 15212, 15309, 15327, 55–40, Iqbal-2000, 16230, 16264, 16281, 16284, 16286, 16002, 16007, 16012, 16027, 16050, 16057, 16081, 16119, 16120, 16133, 16141, 16148, 16149, 16150, 16154, 16163, 16164, 17156, 17160, 17164, 17166, 17167, 17168, 17172, 17178, 17179, 17188, 16097, 16098, 16114
2–3	28	15235, 27–11, 60–57, 80–34, 15100, Uqab-2000, 16234, 16270, 16288, 16034, 16052, 16058, 16060, 16063, 16066, 16080, 16136, 16140, 16155, 16158, 16161, 17151, 17152, 17173, 17174, 17187, 16102, 16115
3–5	27	15153, 15168, 15174, 9408, 16–1154, 13FJ 20, 13FJ 29, NR 520, NR 529, SUPER KAUZ, Annaj-17, AAS-11, Fsd-08, Lasani-08, Pasban-90, Blue Silver, 16262, 16033, 16061, 16065, 16084, 17185, 17189, 17196, 16094, 16104, 16117.
6–10	14	12304, 14116, 14BT 016, PBW 343, SERI, Pb-11, AARI-11, Millat-11, SA-75, 16297, 16055, 17184, 16093, 16100.
11–15	07	JOUHAR-16, Shafaq-06, Parwaz-94, SH-88, Pak-81, Lyp-73, 16009.
16–20	06	Morocco, Seher-06, MH-97, Inq-91, 16278, 16056.
Above 20	02	Morocco, Galaxy-13.
AUDPC/Day Value	No. of genotypes	Genotypes
0	120	60–5, 15082, 15099, 16005, 15113, 15291, 15166, 15216, 1038, 14058, 14061, 20–6, 20–19, 55–33, NS-76, 15–29, 1432, 1578, 1579, 1581, 15–1711, 15–1713, 15–1725, 15–1755, 16-CO38, 16-CO39, NR-521, NR-523, NR-525, 15 BT 001, NW-2-17, Morocco, Ujala-16, Chak-50, Pb-76, Pavon-76, 16222, 16227, 16233, 16259, 16261, 16266, 16274, 16275, 16276, 16277, 16287, 16289, 16282, 16280, 16265, 16290, 16291, 16293, 16294, 16295, 16221, 16260, 16003, 16004, 16005, 16006, 16018, 16023, 16024, 16025, 16036, 16049, 16051, 16077, 16079, 16087, 16090, 16124, 16125, 16128, 16129, 16131, 16132, 16134, 16144, 16145, 16146, 16147, 16152, 16153, 16157, 16150, 16160, 17153, 17154, 17155, 17157, 17158, 17159, 17161, 17162, 17163, 17165, 17169, 17170, 17171, 17175, 17176, 17177, 17180, 17182, 17183, 16106, 16108, 16111, 15012, 15009, 5011, 15018, 15035, 15006, 14003, 14011, 14035.
1–2	43	14124, 14154, 15070, 15212, 15309, 15327, 55–40, Iqbal-2000, 16230, 16264, 16281, 16284, 16286, 16002, 16007, 16012, 16027, 16050, 16057, 16081, 16119, 16120, 16133, 16141, 16148, 16149, 16150, 16154, 16163, 16164, 17156, 17160, 17164, 17166, 17167, 17168, 17172, 17178, 17179, 17188, 16097, 16098, 16114
2–3	28	15235, 27–11, 60–57, 80–34, 15100, Uqab-2000, 16234, 16270, 16288, 16034, 16052, 16058, 16060, 16063, 16066, 16080, 16136, 16140, 16155, 16158, 16161, 17151, 17152, 17173, 17174, 17187, 16102, 16115
3–5	27	15153, 15168, 15174, 9408, 16–1154, 13FJ 20, 13FJ 29, NR 520, NR 529, SUPER KAUZ, Annaj-17, AAS-11, Fsd-08, Lasani-08, Pasban-90, Blue Silver, 16262, 16033, 16061, 16065, 16084, 17185, 17189, 17196, 16094, 16104, 16117.
6–10	14	12304, 14116, 14BT 016, PBW 343, SERI, Pb-11, AARI-11, Millat-11, SA-75, 16297, 16055, 17184, 16093, 16100.
11–15	07	JOUHAR-16, Shafaq-06, Parwaz-94, SH-88, Pak-81, Lyp-73, 16009.
16–20	06	Morocco, Seher-06, MH-97, Inq-91, 16278, 16056.
Above 20	02	Morocco, Galaxy-13.

## Conclusion

The experimental material showing wider range of diversity was evaluated in different agro-ecological zones having variation in climatic factors. The material was inoculated by the mixture of inoculum collected from different parts of Punjab and Sindh province during the previous three years. The gene differentials containing leaf rust genes *Lr*-19, *Lr*-26 and *Lr*-31 showed resistance against the leaf rust in different agro-ecological zones of the Punjab. Hence, the breeders can focus on the introgression of these genes into future breeding material. Among the tested advanced lines, V-14154, V-14124 and HYT 60–5 were very useful advanced lines for release as a commercial variety or use as a parent for leaf rust resistance as they showed good level of resistance against leaf rust. V-14154 (Akbar-19) has been released as a commercial cultivar on the basis of its higher yield, adaptability and disease resistance. Among the current commercial varieties of the Punjab, Ujala-16 has shown the best resistance for leaf rust during study years.
